# Application of Evidence-Based Nursing Intervention in the Treatment of Advanced Squamous Cell Carcinoma of the Lung by Erlotinib Combined with Tegafur, Gimeracil, and Oteracil Potassium and Its Influence on Quality of Life

**DOI:** 10.1155/2021/6801779

**Published:** 2021-12-13

**Authors:** Shan Liu, Xiaocheng Huang, Jin Wen, Fangfang Fu, Huifen Wang

**Affiliations:** ^1^Department of Nursing, Hubei Cancer Hospital, Wuhan 430079, Hubei, China; ^2^Department of Chest Oncology, Hubei Cancer Hospital, Wuhan 430079, Hubei, China

## Abstract

**Objective:**

To explore the application of evidence-based nursing intervention in the treatment of advanced squamous cell carcinoma of the lung by erlotinib combined with tegafur, gimeracil, and oteracil potassium (TS-1) and its influence on quality of life (QOL).

**Methods:**

Clinical data of 92 patients with advanced squamous cell carcinoma of the lung treated with erlotinib and TS-1 in our hospital (January 2017–January 2021) were retrospectively analyzed. Forty-six patients receiving conventional nursing were set as the control group (CG), and other 46 patients receiving evidence-based nursing intervention additionally were set as the study group (SG). The clinical observation indexes of the two groups were compared and analyzed.

**Results:**

No obvious difference in general data between both groups (*P* > 0.05). According to EORTC QLQ-C30, compared with the CG, the scores of role function, physical function, social function, cognitive function, and emotional function in the SG were remarkably higher (*P* < 0.05). After intervention, scores of VAS of patients were obviously lower than those before intervention (*P* < 0.05), and scores of VAS in the SG after intervention were obviously lower than those in the CG (*P* < 0.05). After intervention, scores of SAS and SDS were lower than those before intervention, and those of the SG were obviously lower than those of the SG (*P* < 0.05). Compared with the CG, incidences of adverse reactions such as diarrhoea, nausea and vomiting, erythra, pressure sores, and leukopenia in the SG were obviously lower (*P* < 0.05). Compared with the CG, “very satisfied” and total satisfaction in the SG were obviously higher (*P* < 0.05).

**Conclusion:**

Application of evidence-based nursing intervention in the treatment of advanced squamous cell carcinoma of the lung by erlotinib combined with TS-1 can help patients to relieve pain, improve their psychological state, reduce the incidence of adverse reactions, significantly improve the QOL, and also enhance the satisfaction of clinical nursing.

## 1. Introduction

Squamous cell carcinoma of the lung is one of the nonsmall cell lung cancers (NSCLC) and the most common type of lung cancer, with the incidence and the mortality ranking the first among lung cancers in China [1–3]. According to TNM stages, stage IV is the advanced stage of the disease, and patients have pleural metastasis, pleural effusion, and multiple metastases (liver, brain, bone, etc.). The combined chemotherapy is usually served as the conservative scheme in clinical application to relieve symptoms, enhance survival rate, and improve the quality of life (QOL) [4–7]. Erlotinib is a third-line drug, which is suitable for locally advanced or metastatic NSCLC that two or more chemotherapy regimens fail to work on. Tegafur, gimeracil, and oteracil potassium (TS-1), an oral anticancer agent of fluorouracil derivative, is commonly used in the treatment of NSCLC [5, 8, 9]. Erlotinib combined with TS-1 was implemented in our hospital for patients with advanced squamous cell carcinoma of the lung, which has achieved high disease control rate (DCR). In order to further improve the QOL of patients, our hospital actively explored the nursing intervention that can ensure the prognosis of patients. Currently, symptomatic nursing is the crux for patients with squamous cell carcinoma of the lung; in this way, it should pay more attention to the holistic nursing considering the actual situation of patients. Therefore, evidence-based nursing takes valuable, credible, and scientific research results as the evidence and establishes the nursing concept of guiding and improving practice by research. However, less clinical data are available in patients with advanced squamous cell carcinoma of the lung. Based on the above, this paper will explore the application of evidence-based intervention in the treatment of advanced squamous cell carcinoma of the lung by erlotinib and TS-1 and its influence on QOL, so as to promote the QOL in such patients in the treatment of advanced disease.

## 2. Methods

### 2.1. Screening and Grouping of Patients

Clinical data of 92 patients with advanced squamous cell carcinoma of the lung treated with erlotinib and TS-1 in our hospital (January 2017–January 2021) were retrospectively analyzed. Forty-six patients receiving conventional nursing were set as the control group (CG), and other 46 patients receiving evidence-based nursing intervention additionally were set as the study group (SG). The study was approved and supervised by the Hospital Ethics Committee.

### 2.2. Inclusion Criteria

(1) Patients were diagnosed with advanced squamous cell carcinoma of the lung after pathological examination. (2) According to TNM stages, patients were evaluated as the stage IV. (3) Patients were in line with the indications of the treatment by erlotinib combined with TS-1. (4) The expected survival period was more than 3 months. (5) Patients and their families understood the purpose and the process of the study and signed for the consent form.

### 2.3. Exclusion Criteria

(1) Patients were complicated with other severe organ and tissue pathological changes. (2) Patients were complicated with hematological diseases. (3) Patients had poor treatment compliance or withdrew halfway. (4) Patients had cognitive impairment or could not be communicated with. (5) Patients were pregnant or lactating.

### 2.4. Methods

All patients were treated with erlotinib combined with TS-1. ① Patients were asked to orally take 150 mg of erlotinib hydrochloride (specification: 150 mg; manufacturer: Shanghai Roche Pharmaceutical Co., Ltd.; NMPA approval No. J20170030) 1 h before or 2 h after meals daily until the presence of disease progression or intolerable toxic reaction. ② Patients were asked to take TS-1 (specification: 50 mg; manufacturer: Jiangsu Hengrui Pharmaceutical Co., Ltd.; NMPA approval No. H20100135) twice a day (after breakfast and dinner) for continuous 28 days as a course of treatment, with an interval of 14 days. The first dosage depended on patients' body surface area (m^2^) by tegafur, i.e., 40 mg for <1.25 m^2^, 50 mg for 1.25–1.5 m^2^, and 60 mg for ≥1.5 m^2^. Patients took the drug until they presented with deterioration or they had no drug tolerance [10–12].

CG: according to the doctor's advice, patients were given conventional clinical nursing measures. Meanwhile, patients' physical signs were closely monitored during the treatment. Analgesic drugs should be given timely for those who had severe pain. Attention was paid to patients' negative emotions, and patients were encouraged to strengthen their confidence in treatment.

SG: patients received evidence-based nursing intervention additionally. ① Evidence-based nursing intervention. The actual situation, values, and wishes of patients should be cleared according to the clinical nursing experience of advanced lung cancer. Meanwhile, the nursing staff should also clarify the common complications, adverse reactions, and prevention measures during chemotherapy according to the clinical research data of squamous cell carcinoma of the lung and formulate scientific and reasonable clinical nursing plan with experience. ② The nursing of complications. According to the clinical research data, the incidence of complications was reduced as much as possible after analyzing the relevant risk factors of advanced squamous cell carcinoma of the lung; in addition, erlotinib might trigger liver function injury, which needed to be prevented and treated during nursing according to the patients' drug administration; the results of the domestic clinical trials showed that the incidence of TS-1-related adverse reactions was 83.78%, mainly 68.47% in the blood system (leukopenia 45.05%, thrombocytopenia 20.72%, mostly decreased I and II degrees), 46.85% in the digestive system (nausea and vomiting 39.64%, diarrhoea 7.21%), and 14.41% in others. So, nursing personnel needed to scientifically evaluate the manifestations of adverse reactions in patients and make good control measures. ③ The nursing of pain. Pain assessment should be performed more often to scientifically analyze the results. Relevant knowledge of pain and drug control was publicized for patients. The nursing staff gave analgesic drugs according to the doctor's instructions and helped the patients to improve their pain threshold by diverting their attention. ④ The nursing of body position. Rash was a common side effect of erlotinib. During daily nursing, the nursing staff helped patients to adjust to comfortable position and remind them to change position frequently to avoid pressure sores and the occurrence of other side effects on skin. ⑤ The nursing of exercise. Appropriate exercise could help patients to quickly improve physical strength and enhance immunity. The nursing staff should map out scientific exercise plan based on the patients' gender, needs, and conditions. ⑥ Psychological nursing. According to the patients' family and educational background, the nursing staff took individualized psychological intervention and communicated with them more frequently, so as to help patients to relieve psychological pressure, reduce negative emotions, and increase confidence. Meanwhile, the nurses encouraged family members to accompany, support, and cooperate to give patients more comforts. ⑦ The nursing of discharge. Patients should follow the guidance of scientific and reasonable medication strictly and were encouraged to maintain a positive attitude. Patients were followed up timely and should see a doctor in time in abnormal situations [13–15].

### 2.5. Observation Indexes

The general data including age, BMI, course of disease, gender, basic diseases, and education degree were counted at admission. The EORTC core QOL questionnaire (QLQ-C30), developed by European Organization for Research and Treatment of Cancer (EORTC), was designed to assess the QOL of cancer patients from different countries. Items 29 and 30 have 7 grades, with 1–7 points, and other items have 4 grades, with 1–4 points. Higher scores indicated higher QOL of patients.

The pain degree was evaluated according to Visual Analogue Scale (VAS). 0 points indicated painlessness, and 10 points indicated the most severe pain. Self-Rating Anxiety Scale (SAS) and Self-Rating Depression Scale (SDS) were used to evaluate the psychological changes of patients. The higher the score, the more serious the psychological problems of patients. The self-made nursing satisfaction questionnaire was used to evaluate the patients' satisfaction, which divided into “dissatisfied,” “satisfied,” and “very satisfied.” Total satisfaction = (satisfied + very satisfied)/total × 100%. The Cronbach's *α* coefficient of the scale is 0.935, and the coefficients of other five aspects are within 0.701–0.844, presenting good internal consistency reliability, content validity, and criterion validity. All kinds of adverse reactions of patients were recorded in detail during nursing intervention.

### 2.6. Statistical Processing

All statistical data of the study were processed by SPSS22.0 to calculate the difference between groups, and the pictures were graphed by GraphPad Prism 7 (GraphPad Software, San Diego, USA). Including enumeration data and measurement data in the form of [*n* (%)] and ($\bar{x}$ ± *s*), respectively, the study used *x*^2^ test and *t*-test. The differences were statistically significant at *P* < 0.05.

## 3. Results

### 3.1. General Data

No obvious difference was found between both groups in general data such as age, BMI, course of disease, gender, basic diseases, and education degree (*P* > 0.05), see Table 1.

### 3.2. QOL

According to EORTC QLQ-C30, compared with the CG, the scores of role function, physical function, social function, cognitive function, and emotional function in the SG were remarkably higher (*P* < 0.05), see Figure 1.

The scores of role function, physical function, social function, cognitive function, and emotional function in the CG were (67.81 ± 9.73), (67.83 ± 9.61), (63.11 ± 8.52), (79.03 ± 10.88), and (71.76 ± 9.11) points.

The scores of role function, physical function, social function, cognitive function, and emotional function in the SG were (75.05 ± 10.24), (75.95 ± 10.11), (71.03 ± 9.67), (84.13 ± 9.32), and (80.07 ± 10.05) points.

^*∗*^indicates conspicuous differences in the scores of role function, physical function, social function, cognitive function, and emotional function between both groups from left to right (*t* = 3.476, *t* = 3.948, *t* = 4.168, *t* = 2.414, *t* = 4.155, *P* < 0.05).

### 3.3. Scores of VAS

After intervention, scores of VAS of patients were obviously lower than those before intervention (*P* < 0.05), and scores of VAS in the SG after intervention were obviously lower than those of the CG (*P* < 0.05), see Table 2.

### 3.4. Mental State

After intervention, scores of SAS and SDS were lower than those before intervention, and those of the SG were obviously lower than those of the CG (*P* < 0.05), see Table 3.

### 3.5. Adverse Reactions

Compared with the CG, incidences of adverse reactions such as diarrhoea, nausea and vomiting, erythra, pressure sores, and leukopenia in the SG were obviously lower (*P* < 0.05), see Table 4.

### 3.6. Nursing Satisfaction

Compared with the CG, “very satisfied” and total satisfaction in the SG were obviously higher (*P* < 0.05), see Figure 2.

In the CG, 16 cases were very satisfied, 17 cases were satisfied, and 13 cases were dissatisfied, with the total satisfaction of 33 cases.

In the SG, 26 cases were very satisfied, 18 cases were satisfied, and 2 cases were dissatisfied, with the total satisfaction of 44 cases.

^*∗*^indicates the conspicuous difference in “very satisfied” between the two groups (*X*^2^ = 4.381, *P*=0.036).

^*∗∗*^indicates the conspicuous difference in the total satisfaction between the two groups (*X*^2^ = 9.638, *P*=0.002).

## 4. Discussion

Due to slow growth and late metastases of quamous cell carcinoma of the lung, it is much available to perform surgical resection at the early stage. However, the sensitivity of the cancer to chemoradiotherapy is greatly reduced at the advanced stage, which results in poor treatment effect. Erlotinib and TS-1 are commonly used in the treatment of NSCLC. As a third-line drug, erlotinib can inhibit the intracellular tyrosine phosphorylation related to EGFR, which is commonly used for locally advanced or metastatic NSCLC that two or more chemotherapy regimens fail to work on. While TS-1, with low toxicity, can inhibit the phosphorylation of 5-fluorouracil (5-Fu), reduce toxicity of 5-Fu, maintain higher drug concentration in plasma, and improve anticancer activity [16–19]. Therefore, this treatment method was applied in patients who were in line with the indications of the treatment by erlotinib combined with TS-1 in this study, which achieved higher DCR. After first-line and second-line treatment, the QOL of patients with advanced squamous cell carcinoma of the lung is seriously reduced due to various pains, adverse reactions of chemotherapy, and psychological pressure, which is much of great distress for patients.

In order to ensure the treatment effect, it has always been the focus of clinical research to explore the nursing intervention suitable for patients with advanced squamous cell carcinoma of the lung. Evidence-based nursing intervention is a new nursing concept under the guidance of evidence-based medicine, which means that nurses should combine the recent research results of diseases with clinical nursing experience and patients' subjective will in the nursing process and then formulate a scientific and reasonable individualized nursing program, so as to provide patients with better nursing measures and comprehensively improve their QOL. This mode puts more emphasis on scientific and planned nursing intervention rather than that only conforming to doctor's advice, which has improved efficacy of clinical nursing [15, 20–22]. With the intervention of evidence-based medicine, the evidence-based nursing intervention provided a more scientific protection for the combined treatment of erlotinib and TS-1. Under the guidance of evidence-based medicine combined with patients' wishes, the disease characteristics of patients with advanced squamous cell carcinoma of the lung were comprehensively analyzed, and individualized evidence-based intervention program was formulated, which was recognized by patients. Therefore, this paper retrospectively analyzed the clinical data of some patients in order to establish a developed and scientific nursing program for patients.

After intervention, scores of VAS of patients were obviously lower than those before intervention (*P* < 0.05), and scores of VAS in the SG after intervention were obviously lower than those in the CG (*P* < 0.05). It indicated that the evidence-based nursing intervention had better efficacy of relieving pain for patients, which was also in line with the results of the study of Korhonen [23]. After intervention, scores of SAS and SDS were lower than those before intervention, and those of the SG were obviously lower than those of the CG (*P* < 0.05). After a series of treatment failure, many patients with advanced squamous cell carcinoma of the lung suffer from severe depression, anxiety, and fear of adverse reactions. Therefore, application of evidence-based nursing is more effective in psychological intervention and helpful to change the psychological mood of patients and increase the confidence of treatment. Compared with the CG, incidences of adverse reactions such as diarrhoea, nausea and vomiting, erythra, pressure sores, and leukopenia in the SG were obviously lower (*P* < 0.05), demonstrating that evidence-based nursing intervention paid much attention to preventive measures of adverse reactions, which could better relieve physical and psychological distress for patients. According to EORTC QLQ-C30, compared with the CG, the scores of role function, physical function, social function, cognitive function, and emotional function in the SG were remarkably higher (*P* < 0.05). Compared with the CG, “very satisfied” and total satisfaction in the SG were obviously higher (*P* < 0.05). It indicated evidence-based nursing intervention could better improve QOL of patients than conventional nursing, which was supported and recognized by patients.

To sum up, application of evidence-based nursing intervention in the treatment of advanced squamous cell carcinoma of the lung by erlotinib combined with TS-1 can help patients to relieve pain, improve their psychological state, reduce the incidence of adverse reactions, significantly improve the QOL, and also enhance the satisfaction of clinical nursing. The disadvantage of this study was that it was a single-center study with small sample, which needed to be confirmed by expanding the sample size and carrying out multicenter studies; in addition, the study objects were mainly patients in the advanced stage, but the prognosis follow-up time was short and analysis about patients' survival was not involved, so its extended exploration value is high, and subsequent in-depth study can be conducted.

## Figures and Tables

**Figure 1:** Comparison of scores of EORTC QLQ-C30. Note: the abscissa was the evaluation dimensions, including role function, physical function, social function, cognitive function, and emotional function, and the ordinate was the score, points.

**Figure 2:** Comparison of nursing satisfaction. Note: the abscissa indicated evaluation dimensions, and the ordinate indicated the percentage (%).

**Table 1:** Comparison of general data (*n* = 46).

Observation indexes	CG	SG	*t*/*X*^2^	*P* value
Age (years old)	59.24 ± 8.76	58.85 ± 8.92	0.212	0.833
BMI (kg/m^2^)	23.21 ± 3.15	23.34 ± 3.22	0.196	0.845
Course of disease (years)	4.46 ± 1.03	4.39 ± 1.01	0.329	0.743
Gender			0.177	0.674
Male	27 (58.70)	25 (54.35)		
Female	19 (41.30)	21 (45.65)		
Basic diseases				
Diabetes	23 (50)	20 (43.48)	0.393	0.531
Hypertension	18 (39.13)	19 (41.30)	0.045	0.832
Hyperlipemia	13 (28.26)	15 (32.61)	0.205	0.650
Education degree			0.192	0.662
High school degree below	31 (67.39)	29 (63.04)		
Junior high school degree and above	15 (32.61)	17 (36.96)		

**Table 2:** Comparison of scores of VAS.

Group	*n*	Before intervention	After intervention
CG	46	6.45 ± 1.35	5.88 ± 1.05^*∗*^
SG	46	6.52 ± 1.42	5.16 ± 1.12^*∗*^
*t*		0.242	3.181
*P* value		0.809	0.002

Note: ^*∗*^indicates *P* < 0.05 in the comparison of VAS scores before and after intervention in each group.

**Table 3:** Comparison of scores of SAS and SDS.

Group	SAS		SDS	
	Before intervention	After intervention	Before intervention	After intervention
CG	59.14 ± 8.75	47.85 ± 7.14^*∗*^	62.07 ± 9.43	48.57 ± 9.10^*∗*^
SG	58.27 ± 8.82	42.03 ± 7.26^*∗*^	61.89 ± 9.33	44.26 ± 8.70^*∗*^
*t*		3.876		2.322
*P* value		<0.001		0.023

Note: ^*∗*^indicates significant differences in scores before and after intervention in each group (*P* < 0.05).

**Table 4:** Comparison of adverse reactions.

Group	*n*	Diarrhoea	Nausea and vomiting	Erythra	Pressure sores	Leukopenia
CG	46	16 (34.78)	6 (13.04)	17 (36.96)	5 (10.87)	13 (28.26)
SG	46	7 (15.22)	1 (2.17)	5 (10.87)	0 (0)	3 (6.52)
*X* ^2^		4.696	3.866	8.603	5.287	7.566
*P* value		0.030	0.049	0.003	0.021	0.006

## Data Availability

The data used to support the findings of this study are available on reasonable request from the corresponding author.
